# Prediction of Metabolic Characteristics of Cardiovascular and Cerebrovascular Diseases Based on Convolutional Neural Network

**DOI:** 10.1155/2022/3206378

**Published:** 2022-07-27

**Authors:** Zhengfei Yang, Ping Li, Rui Wang

**Affiliations:** ^1^Institute of Traditional Chinese Medicine, Ningxia Medical University, Yinchuan 750000, China; ^2^Weifang Engineering Vocational University, Weifang, Shandong Province, 262500, China

## Abstract

As a typical disease, cardiovascular and cerebrovascular diseases cause great damage to the human body. In view of the problem that the existing models failed to describe and represent the characteristics of cardiovascular and cerebrovascular indicators, convolution neural network was used to analyze the metabolic factors of cardiovascular and cerebrovascular. Based on convolutional neural network theory, feature extraction was carried out on the relevant parameters of the model, and the change trend of different cardiovascular and cerebrovascular indicators was studied by model optimization, theoretical analysis, and experimental verification. Relevant studies show that the value of neurons increases slowly at first and then rapidly with the increase of bias term *b*. And with the increase of computing time, the corresponding nonlinear characteristics are gradually reflected; so, the influence of computing time on neuron results should be considered when selecting bias term *b*. The gradient changes under different functions have typical symmetry, which indicates that the effects of functions on model parameters have certain cyclic characteristics. Among them, ReLU function has the largest variation range, tanh function has a relatively small curve variation range, and sigmoid function has the smallest variation range. Five indicators are selected to describe the metabolic characteristics of the disease through characteristic analysis of cardiovascular and cerebrovascular diseases. The onset signs have the greatest impact on cardiovascular and cerebrovascular diseases, while the corresponding metabolic characteristics have the least impact on cardiovascular and cerebrovascular diseases. The study showed that the influence of different indicators on the model had typical stage characteristics, and relevant data were used to verify the accuracy of the model. Finally, the optimization model based on convolutional neural network was used to predict the metabolic characteristics of cardiovascular and cerebrovascular diseases. Relevant studies show that the optimization model can better analyze the metabolic characteristics of cardiovascular and cerebrovascular diseases. This research can provide theoretical support for the application of convolutional neural networks in other fields.

## 1. Introduction

Convolutional neural network has a wide application prospect in different fields, and its application directions mainly include video anomaly detection [1], vehicle tracking [2], photovoltaic product detection [3], lime structure calculation [4], and high-speed train [5]. In view of the low accuracy of robust time series, the optimization model under convolutional neural network was used to conduct a targeted analysis of genetic algorithm [6]. First, the characteristic parameters of the model were extracted. The corresponding optimization parameters were obtained by parameter extraction, and then the model features in the time series parameters were further modified to obtain the optimization algorithm that can characterize the model sequence. Finally, the accuracy of the model was verified by relevant experimental data. In view of the problems existing in the original convolutional neural network model in the study of prostate cancer and other symptoms, the revised convolutional neural network model was adopted to further analyze the data of relevant symptoms [7], so as to obtain the corresponding optimization results, which can be verified by the model. In biomedicine, based on the relevant theories of convolutional neural network, the feature insertion method was adopted to analyze the relevant features of organisms [8], and the corresponding optimization results were finally obtained. Finally, relevant data was used to prove the model.

The above studies mainly focus on the application of convolutional neural network in engineering and other aspects, but there were relatively few studies on cardiovascular and cerebrovascular diseases; so, it was necessary to carry out studies on the metabolic characteristics of cardiovascular and cerebrovascular diseases. Based on the relevant theory of convolutional neural network, this paper conducts targeted research on the related problems in cardiovascular and cerebrovascular diseases by means of feature extraction, model insertion, and experimental verification. Studies have found that different indicators can describe metabolic characteristics of cardiovascular and cerebrovascular diseases, indicating that the correlation optimization model based on convolutional neural network can carry out correlation analysis and prediction of metabolic characteristics of cardiovascular and cerebrovascular diseases, and provide support for the application of convolutional neural network in different fields.

## 2. Basic Theory of Convolutional Neural Networks

The genetic algorithm is a kind of random search algorithm, which regards a biological individual as a solution in the optimization algorithm, and the population composed of many individuals is the solution set of the algorithm [9, 10]. Then, through genetic operations such as selection crossover and mutation of the population, the poor individuals are constantly eliminated, and the individual genes with favorable mutation are passed on to the next generation through probabilistic selection, after continuous iteration and update. When the termination condition is reached, the output individual is the optimal one that survives after screening. The genetic algorithm is easy to operate and can be applied to both continuous optimization problems and discrete problems. Its multidirection global optimization performance has a good theoretical value for solving complex optimization problems today.

### 2.1. Basic Knowledge of Neural Network

Machine learning, as one of the ways to achieve artificial intelligence, has been revived in recent years with the development of high-performance computer hardware such as image processors and mobile Internet [11, 12]. Deep learning is a kind of nonlinear neural network with multiple hidden layers. It imitates the working mechanism of human brain neurons and constantly extracts features for learning and analysis under the training of a large amount of data. It has strong generalization. It has been widely used in machine vision, natural language processing, autodriving, semantics, speech recognition, and other fields.

Traditional learning model and deep learning model have many shortcomings in theoretical practice and relevant calculation methods. Deep learning is using more data or better algorithms to improve the results of a learning algorithm. For some applications, deep learning works better on large data sets than other machine learning methods. Moreover, deep learning is more suitable for unlabeled data; so, it is not limited to the field of natural language processing mainly based on entity recognition. In order to further illustrate the differences between the two models, we drew the model performance curves of the traditional learning model and the deep learning model based on relevant experimental data, as shown in Figure 1. It can be seen from the figure that with the continuous increase of data, the performance of corresponding curves shows different trends. From the perspective of traditional learning model, this model has typical two-stage characteristics. In the first stage, with the gradual increase of test data, the corresponding model performance values show a gradually increasing trend, but the slope of the increasing curve gradually decreases. When the corresponding data reaches 75 or so, the slope of the corresponding curve is zero. When it exceeds 75, the model performance data of the corresponding traditional learning model shows a constant change trend with the gradual increase of data, indicating that the gradual increase of data has no influence on the model performance. The curve of the deep learning model can be divided into three stages according to the different characteristics of changes. In the first stage, the curve shows a slow rise. With the gradual increase of data, the corresponding model performance parameters gradually improve, and the corresponding curve slope also shows a trend of slow decline. However, the slope of the corresponding curve is higher than that of the traditional learning model of the same period. The second stage of the curve is the stage of steady increase, in which the slope of the corresponding curve shows an approximately constant trend, indicating that the model performance of this stage gradually improves with the increase of data. When it exceeds the critical value of the second stage, the curve enters the third stage. In the third stage, the performance of the deep learning model gradually improves with the increase of experimental data, and the slope of the corresponding curve increases rapidly. This indicates that the slope of the curve shows a typical nonlinear increasing trend at this stage. Therefore, it can be seen from the above analysis that the deep learning model can describe two stages of nonlinear increase and nonlinear attenuation, while the traditional model can only describe the nonlinear attenuation stage and cannot give a good description of the nonlinear acceleration stage.

Artificial neural network (ANN) is a kind of neural network that simulates the process from activation to signal sending of brain neurons and organizes many neurons according to certain hierarchical structure to form multilayer neural network [13, 14]. At first, the neural network in biology was abstracted into a simple linear model based on threshold logic algorithm, called MP (McCulloch-Pitts) neuron model. The MP neuron model has a wide range of applications in different fields. The MP neuron model has the following capabilities: (1) Each neuron is an information processing unit with multiple inputs and single outputs; (2) Neuron input can be divided into excitatory input and inhibitory input. (3) Neurons have spatial integration characteristics and threshold characteristics. (4) There is a fixed time delay between the input and output of neurons, mainly due to synaptic delay.

It can be seen from the above analysis that the MP model, as one of the convolution neural network models, can calculate different types of data. In order to analyze the calculation principle of this MP model, the corresponding MP model is summarized as shown in Figure 2. It can be seen from the figure that the calculation of MP model first requires crossreplacement of different types of data corresponding to *x* and *w*, so that the corresponding data can have typical characteristics. Then, these representative parameters are imported into the corresponding *b* module, through which parameters are extracted, analyzed, and optimized, so that the obtained neuron data can further reflect the optimal value and corresponding parameter characteristics of the *b* model. Then, the obtained parameter characteristics are further calculated and output. Finally, the optimized data are further verified by the targeted model verification method, and finally, the optimized model data is output.

Corresponding neurons can be expressed as follows:

(1) $$\begin{array}{c} y_{i}=f\times \left(\underset{i}{\sum }w_{i}x_{i}+b\right), \end{array}$$

where (*x*_1_, *x*_2_, *x*_3__,_…, *x*_*n*_) and (*y*_1_, *y*_2_, *y*_3_,…, *y*_*n*_) are the input and output values of the network, respectively. *I* represents the input or output of the *i*-th neuron, (*w*_1_, *w*_2_, *w*_3_,…, *w*_*n*_) is the connection weight value of the network, and *b* is the bias term.

In order to further analyze the influence of bias term *b* on neuron parameters, we obtained the corresponding neuron calculation data according to the calculation formula and theory of bias term *b* and obtained the contour diagram of neuron changes under the action of bias term *b*, as shown in Figure 3. It can be seen from the figure that with the increase of bias term *b*, the corresponding neuron value increases slowly at first, and then when the bias term *b* reaches about 20, the corresponding curve shows a rapid increase trend, and the corresponding slope also shows a nonlinear increase. When the bias term *b* exceeds about 27, the slope of the corresponding curve drops rapidly, indicating that the effect of bias term *b* on neuron parameters has typical nonlinear characteristics. Therefore, it is necessary to comprehensively consider the variation range of bias term b in computational neurons, so as to obtain accurate computational parameters of neurons.

Activation function is an indispensable nonlinear mapping function in convolutional neural network. The use of activation function in neural network is equivalent to introducing nonlinear factors into neurons, so that they have nonlinear fitting ability and can be applied to various nonlinear models and increase the richness of neural network expression ability.

The sigmoid logic function is the earliest and most commonly used activation function. The corresponding function expression is as follows:

(2) $$\begin{array}{c} \text{sigmoid}\left(x\right)=\frac{1}{1+e^{-x}}. \end{array}$$

Tanh function is the deformation of the above functions, and the mathematical expression is as follows:

(3) $$\begin{array}{c} \tanh\left(x\right)=\frac{e^{x}-e^{-x}}{e^{x}+e^{‐x}}. \end{array}$$

The curves of tanh function and sigmoid function are very similar. The difference is that the output interval expands from (0, 1) to (-1, 1), and zero is taken as the output center.

ReLU activation function is also called modified linear unit, and the formula is as follows:

(4) $$\begin{array}{c} \text{f}\left(\text{x}\right)=\left\{\begin{array}{c} x,x\geq 0,\\ 0,x<0. \end{array}\right. \end{array}$$

ReLU is a piecewise linear function that can prevent some neurons from being activated, thus enhancing the sparsity and learning accuracy of the network and avoiding the overfitting phenomenon. When the input value is positive, only linear operation is needed, the calculation speed and convergence speed are much faster than the above two functions, and the problem of gradient disappearance is solved.

Through the above formula and theoretical analysis, it can be seen that different functions have different trends of change. In order to qualitatively analyze this change trend, we use gradient graph to analyze three different functions and draw corresponding gradient graph under different functions. The specific change curve is shown in Figure 4. It can be seen from the figure that three different functions have three different changing trends. However, it can be seen from the figure that the three different functions have typical symmetric characteristics, and the axis of symmetry is *x* = 0. It can be seen from the sigmoid function that, with the gradual increase of parameter *x*, the corresponding *y* value first presents a slow increase trend, and the corresponding slope also presents a gradual increase change. When it reaches the highest point, the corresponding *y* value is only 0.24. When it exceeds the maximum value, the corresponding curve declines gradually, and the slope also shows a trend of gradually approaching zero. It can be seen from the curve of tanh function that in the first stage, the curve shows a slow and approximately constant change, while when *x* is -2, the corresponding curve increases rapidly. The slope of the corresponding curve also shows a nonlinear increasing trend. When it reaches the maximum value of 0.95, the corresponding *x* is also 0. When the curve exceeds the highest point, the corresponding curve shows a rapid decline. From the change curve of ReLU function, we can see that the corresponding curve shows a change trend parallel to the *y*-axis. Through the above analysis, we can see that the curves corresponding to three different functions have different characteristics of change; so, we need to analyze the specific situation qualitatively and then select different functions to solve and verify the parameters.

### 2.2. Convolutional Neural Network

Convolutional neural network is a kind of multilayer feedforward neural network, which is also one of the important forms of deep neural network [15, 16]. It is specially used to process data with network topology.

Convolutional neural network models have different changing characteristics in the process of calculation and development. In order to further analyze convolutional neural network models, the corresponding development flow chart is obtained by summarizing the development history of some models, as shown in Figure 5. It can be seen from the figure that the convolutional neural network model can be divided into four different types of variable modules: first, new functional unit modules are added, which can further improve the calculation accuracy and operation range of the model. The second is to make a breakthrough from two aspects of detection and classification. The third is to enhance the relevant functions of the convolution module and improve the operation effect of the corresponding model. Fourth, network deepening is carried out for the model.

The convolution layer of the convolutional neural network is composed of one or more convolution kernels and feature graphs [17, 18]. The size of the convolution kernel is usually odd, and the features of the feature graph of the upper layer are extracted through the convolution operation of the convolution kernel to output the feature graph of the next layer. The specific calculation formula is as follows:

(5) $$\begin{array}{c} N=\frac{W‐F+2\text{P}}{S}+1, \end{array}$$

where *N* is the size of the output image, *W* is the size of the input image, *F* is the size of the convolution kernel, *P* is the filling number of the image edge, and *S* is the sliding step. The influence of sliding steps *S* on the convolution kernel in the convolutional neural network is mainly reflected in the following aspects: The larger the moving step *S* of the sliding window is, the smaller the size of the output feature graph is, and the fewer image features it carries.

Through the above analysis, it can be seen that the convolution layer is composed of parameters of different types and characteristics, among which the most influential ones are input image size *W*, convolution size *F*, image filling edge *P*, and step size *S*. In order to further analyze the specific rules of the size of the output image, the change curves of the size of the convolution running image under different parameters are drawn, as shown in Figure 6. It can be seen from the figure that with the gradual increase of the size value, the corresponding curve has typical nonlinearity and diversity. As can be seen from the change process of parameter *W*, with the gradual increase of graph size value, the corresponding curve first presents a slow increase trend. Then, when the size value is 825, the corresponding curve drops rapidly to the lowest value. When the curve reaches the lowest point, the curve rises rapidly with an approximate constant slope, and then the corresponding curve shows a gentle change when it immediately reaches the local maximum value. It can be seen from the change curve of parameter *F* that with the gradual increase of size value, the corresponding curve increases rapidly, and the slope also reaches the maximum value and then gradually decreases. When it reaches the lowest value, the curve gradually tends to be gentle with the increase of the size, which indicates that the influence of parameter *F* on the size of the graph only remains at a relatively low value. It can be seen from the curve change of parameter *P* that with the gradual increase of the size value, the corresponding curve increases rapidly first, but the slope of the curve is lower than that of the corresponding parameter *F*. When it reaches the maximum value, the curve also shows a downward trend, but the corresponding downward value is also less than the parameter *F* and then tends to gentle. It can be seen from the curve corresponding to *S* value that the overall trend of the curve of this parameter is basically the same as that of the curve of parameter *P*, except that the specific value is slightly different. Therefore, it can be seen that the curves of parameters *F*, *P*, and *S* have obvious variation characteristics: In other words, the corresponding influence is more obvious in the small size, and with the gradual increase of size, the corresponding calculation value of size output is more constant. Therefore, through comprehensive consideration, we can see that the corresponding output image size *W* has the greatest influence on the convolution layer.

The corresponding operation formula of the convolution layer of the convolutional neural network is shown as follows:

(6) $$\begin{array}{c} f\left[x,y\right]*g\left[x,y\right]=\overset{a}{\underset{n_{1}=‐\text{a}}{\sum }}\overset{a}{\underset{n_{2}=‐a}{\sum }}f\left[n_{1},n_{2}\right]\times g\left[x-n_{1},y-n_{2}\right], \end{array}$$

where *f*[*n*_1_, *n*_2_] is the input image, *g*[*n*_1_, *n*_2_] is the convolution kernel, and *n*_1_ and *n*_2_ represent pixel points. *P* is the number of parameters of the convolution layer.

Parameter *P* is obtained by multiplying the dimensions of the convolution kernel *K*_*w*_ and *K*_*h*_, the number of input channels *C*_1__,_ and the number of input channels *C*_2_, and the corresponding formula is expressed as

(7) $$\begin{array}{c} P=K_{w}\times K_{h}\times C_{1}\times C_{2}. \end{array}$$

In order to further analyze the influence of size and channel on parameter quantity, the quantitative change diagram of parameter quality under two different parameters was drawn, as shown in Figure 7. It can be seen from the figure that with the increase of parameter *K*, the corresponding curve histogram shows a trend of gradual increase. Especially when parameter *C* is constant at the maximum value, the value of the corresponding parameter *K* increases the most. When the parameter *K* is constant, the curve corresponding to parameter *C* shows an obvious fluctuation trend. This indicates that the influence of parameter *K* on the number of parameters is more obvious, while the influence of parameter *C* on the number of parameters is more volatile. Therefore, it is necessary to comprehensively consider the proportion of parameter *K* and parameter *C* in the specific operation process, so as to obtain the accurate number of parameters. The size of convolution check is mainly represented by parameter *K*, while the corresponding channel is mainly described by the number of input channels *C*. The research methods and contents of the two different parameters are different, resulting in different influences on the convolution parameter *P*.

### 2.3. Parameter Optimization of Convolutional Neural Network

Currently, the main pooling operations are maximum pooling, average pooling, and random pooling [19, 20]. Maximum pooling compares the values of pixels in each region and selects the maximum value within the pixel region as the output of this pixel region. Average pooling takes the average of pixels in each region as the output of the pixel region. Random pooling randomly selects pixels in the region according to their probability as the output of the pixel region, which improves the generalization ability.

After the pooling operation, the output image size calculation formula is as follows:

(8) $$\begin{array}{c} O=\frac{I-P_{s}}{S}+1, \end{array}$$

where *O* is the size of the pooled output image, *I* is the size of the input image, *P*_*s*_ is the size of the pooled layer, and *S* is the moving step. For maximum pooling, the default step is *S* = 2.

In order to further analyze the specific influencing factors of the size of the pooled output image, we drew the output curves of the pooled size image under several different influencing factors, as shown in Figure 8. It can be seen from the curve that the effects of different parameters on the pooling of convolutional neural networks have different performance characteristics. The curve as a whole can be divided into two phases. In the first stage, with the gradual increase of *P*_*s*_ and size output and input values, the corresponding curve shows an approximately constant linear change, while the corresponding parameter *I* shows a linear decline in the first stage, and the slope of the corresponding curve is higher than that of *P*_*s*_. This indicates that in the first stage, the influence of parameter *P*_*s*_ on the output value *O* is higher than that of parameter *I*. And the corresponding curve of the output image size after pooling also shows a trend of gradual decline. In the second stage, as the corresponding parameter *P*_*s*_ increases with the input value, the corresponding size output value shows a trend of gradual decline, while the corresponding parameter *I* curve shows a trend of fluctuation first and then gradually rising. Finally, the data of parameter *O* shows a trend of gradual increase with the increase of the input value.

The full connection layer usually appears at the end of the convolutional neural network. Since the fully connected layer can only accept 2D matrix, it is necessary to convert the 3D feature tensor of the image extracted by the previous convolution layer into a long vector. Then, the full connection layer performs classification or regression tasks. For the output of the *i*-th neuron of layer *L*, the calculation formula of the full connection layer is as follows:

(9) $$\begin{array}{c} x_{i}^{l}=f\left(\overset{n}{\underset{j=1}{\sum }}x_{j}^{l-1}w_{i,j}^{l-1}+b_{i}^{l-1}\right), \end{array}$$

where *x*_*j*_^*l*−1^ is the output value of the *j*-th neuron in layer l-1, *w*_*i*,*j*_^*l*−1^ is the connection weight between the *j*-th neuron in layer l−1 and the *i*-th neuron in layer l, *n* is the number of neurons in layer l −1, and *b*_*i*_^*l*−1^ is the corresponding bias quantity of the *i*-th neuron in layer l.

The sigmoid, also known as the squeeze function, is a very common dichotomy method that squeezes input values that fluctuate over a wide range into an output interval of (0, 1). The advantages of this function are as follows: (1) the function curve is smooth, and (2) the function is continuous everywhere and easy to differentiate. Disadvantages of sigmoid function are as follows: (1) easy to saturate and (2) large amount of calculation, both forward and back propagation involves division and power operation, which increases the training time. The mathematical expression of softmax function is as follows:

(10) $$\begin{array}{c} \text{softmax}\left(z_{i}\right)=\delta \left(z_{i}\right)=\frac{\exp\left(z_{i}\right)}{\sum_{j=1}^{m}\exp\left(z_{i}\right)}, \end{array}$$

(11) $$\begin{array}{c} \text{loss}=\text{ylo}{\text{g}}_{2}^{\hat{y}}, \end{array}$$

where *i* is the node, *j* is the category index, *m* is the number of output nodes, and $\hat{\text{y}}$ is the output predictive value of the neural network for cardio-cerebrovascular. The change of the result of category index *j* will have a great influence on softmax function, and the range of category index *j* is (1, *m*). The sum of all output values of the softmax function is as follows:

(12) $$\begin{array}{c} \overset{j}{\underset{i=0}{\sum }}\delta \left(z_{i}\right)=1. \end{array}$$

The change of parameter *i* will lead to the change of model prediction parameters. In order to further analyze the influence rule of parameter *i* on sample prediction value, the model prediction proportion curves under different parameters are drawn, as shown in Figure 9. As can be seen from the figure, as the number of samples increases gradually, the proportion of the predicted value corresponding to parameter *i* = 1 shows a fluctuating trend of increasing first, then stabilizing and finally increasing again, indicating that parameter *i* = 1 has a great influence on the parameter. The reason is that parameter *i* further affects the proportion of the model by changing the specific value and calculation method of the output function. When parameter *i* = 2, the proportion of the corresponding model shows a trend of gradual increase. When the parameter is increased to 3, the proportion curve of the corresponding model shows a relatively stable trend as the number of samples increases. This indicates that parameter *i* = 3 has a limited influence on the model. Finally, when parameter *i* = 4, the volatility of corresponding model parameters is more obvious than that when parameter *i* = 1. Based on the above analysis, we can see that parameter *i* has different influences on parameters of different samples, and the specific value and basis of parameter sample number should be considered comprehensively in sample analysis. Thus, a clear calculation process and accurate calculation results are obtained.

## 3. Application and Prediction of Convolutional Neural Networks in Cardiovascular and Cerebrovascular Diseases

### 3.1. Main Features of Metabolism of Cardiovascular and Cerebrovascular Diseases

As a relatively common disease, cardiovascular and cerebrovascular diseases do great harm to the human body. In order to further quantitatively analyze the changing rules and characteristics of cardiovascular and cerebrovascular diseases in the metabolic process, five different characteristic parameters are selected to describe the cardiovascular and cerebrovascular diseases. The five characteristic parameters were metabolic characteristics, clinical manifestations, blood circulation, organ senescence, and symptom of disease. As an indirect manifestation of cardiovascular and cerebrovascular diseases, metabolic characteristics can reflect the related characteristics of cardiovascular and cerebrovascular diseases. Therefore, metabolic characteristics of patients need to be analyzed in daily life, so as to obtain more accurate results. As the direct manifestation of cardiovascular and cerebrovascular diseases, clinical manifestations can improve the precise treatment for patients with cardiovascular and cerebrovascular diseases and provide a strong guarantee for the rehabilitation of cardiovascular and cerebrovascular diseases. Blood circulation is a very complex index, which can not only reflect the related content of cardiovascular and cerebrovascular but also judge the physical health of patients through relevant tests. Organ aging is a complication of cardiovascular and cerebrovascular diseases. We can further improve the precision of relevant treatment schemes for cardiovascular and cerebrovascular diseases by delaying organ aging. As an important indicator of cardiovascular and cerebrovascular diseases, symptoms can provide strong guarantee and support for clinical treatment and rehabilitation. Through the statistics and analysis of a large number of clinical data, the characteristic indexes of the influence of different characteristic parameters on cardiovascular and cerebrovascular diseases were obtained, as shown in Figure 10. According to the proportion in the figure, it can be seen that metabolic characteristics have the least influence on cardiovascular and cerebrovascular diseases, only 9.68%. Clinical manifestations accounted for about 13%. The proportion of blood circulation is about 20%. Organ senescence accounted for 25.8%. The proportion of symptoms was the highest, about 32.3%.

### 3.2. Application of Convolutional Neural Network in Metabolic Features of Cardiovascular and Cerebrovascular Diseases

Through the above analysis and research, we can see that convolutional neural network has good application in different fields [21, 22]. In view of the problems related to metabolic characteristics in cardiovascular and cerebrovascular diseases, in order to better analyze the influence of the characteristics of cardiovascular and cerebrovascular diseases on the disease, relevant theories of convolutional neural network are introduced to build the corresponding optimization model. Furthermore, the optimized convolutional neural network model was used to further analyze the metabolic characteristics of cardiovascular and cerebrovascular diseases and to make targeted prediction of cardiovascular and cerebrovascular diseases.

In order to further apply convolutional neural network to metabolic analysis of cardiovascular and cerebrovascular diseases, a calculation method of cardiovascular and cerebrovascular diseases based on convolutional neural network was obtained through model optimization and theoretical analysis. In order to further explain this calculation process accurately, a characteristic flow chart of cardio-cerebrovascular metabolism based on convolutional neural network was drawn, as shown in Figure 11. It can be seen from the figure that the basic parameters of cardiovascular and cerebrovascular diseases need to be set first, and then the metabolic characteristics of cardiovascular and cerebrovascular diseases are analyzed by using the initialization grid in the convolutional neural network and then imported into the pretransmission process. In this way, the related cardiovascular and cerebrovascular characteristic parameters are further elaborated and extracted, and then the calculation process is discriminated by the judgment equation. If it does not meet the relevant requirements, the error calculation and network weight modification shall be carried out, and the obtained results shall be further iterated. Finally, the optimized results shall be imported into the test model for further analysis, and finally, the optimized characteristics of cardiovascular and cerebrovascular diseases shall be derived.

The above methods can be used to further analyze the metabolic characteristics of cardiovascular and cerebrovascular diseases, so as to obtain the corresponding metabolic results and index curves, as shown in Figure 12. From the curve changes in the figure, we can see that metabolic indicators at different steps have different output results, which indicates that the selection of different indicators has a wide range of descriptions, which can be used to describe different aspects of cardiovascular and cerebrovascular diseases. As the number of iterations increases, the metabolic characteristics of cardiovascular and cerebrovascular diseases first show a trend of rapid increase, and the constant slope of the corresponding curve indicates that the change conforms to the change of linear characteristics. However, with the further increase of iteration steps, the corresponding index output value shows a slow increase trend. And the slope is going to be lower than the first step. It can be seen from the clinical performance indicators that the curve has obvious fluctuation characteristics, which firstly drops rapidly to the lowest point, and then shows a slow increase trend with the increase of the number of iterations, indicating that the clinical performance can well describe the linear changes of cardiovascular and cerebrovascular output values at different stages. Blood circulation has a typical symmetry, indicating that its description of cardiovascular and cerebrovascular can have obvious regularity. The blood circulation curve showed a slow decline at first and then a rapid decline to the lowest point, followed by a significant improvement with the increase of iteration steps. The characteristic indexes of organ senescence of cardiovascular and cerebrovascular diseases have a relatively constant change trend under different steps; that is, organ senescence does not change with the change of iterative steps, which is an inherent attribute of cardiovascular and cerebrovascular diseases. The curve of the corresponding symptom increases slowly at first, and with the increase of iteration number, the curve has a significant increase range, indicating that the curve corresponding to the symptom has a significant change to the higher iteration number. The reason for the changes in metabolic indicators of cardiovascular and cerebrovascular diseases is that metabolic characteristic parameters are calculated by different change functions. The obtained results are imported into the convolutional neural network for optimization of corresponding parameters, so that the obtained results have different change characteristics, which can describe different types of cardiovascular and cerebrovascular diseases.

## 4. Discussion

The above analysis carried out targeted analysis on the metabolic characteristics of cardiovascular and cerebrovascular diseases under different indicators, indicating that the metabolic characteristics of cardiovascular and cerebrovascular diseases based on convolutional neural network can well describe the specific conditions of patients with cardiovascular and cerebrovascular diseases. In order to further analyze and predict the changing trend of cardiovascular and cerebrovascular diseases and provide better medical services for patients, convolutional neural network was adopted to analyze the relevant data and indicators of cardiovascular and cerebrovascular diseases, so as to obtain the model prediction curves of cardiovascular and cerebrovascular diseases at different times, as shown in Figure 13. Through the specific changes of the test curve and model curve, it can be seen that the cardio-cerebrovascular indicators based on convolutional neural network can well reflect the real cardio-cerebrovascular data, and there are overlapping indicators in different time periods. This also shows the accuracy of model index selection from another aspect. And it can be seen from the prediction that cardiovascular and cerebrovascular diseases show an obvious trend of improvement with the increase of time. However, when it reaches a certain time, the curve shows a slow decline, which indicates that cardiovascular and cerebrovascular diseases have different characteristics of change at different times. We need to take different measures according to the actual situation to carry out targeted evaluation and evaluation of cardiovascular and cerebrovascular diseases. The selection of the corresponding parameters of cardiovascular and cerebrovascular diseases is uncertain, and the corresponding parameters will show a complex change process with the difference of time and samples, which will lead to the deviation between the calculated results and the actual results.

## 5. Conclusion

1. The traditional learning model is a typical two-stage change feature, which can describe the attenuation and stability stages of characteristic parameters. However, it cannot describe the nonlinear increase stage because it does not consider the factor of nonlinear increase. However, due to the introduction of nonlinear factors, the deep learning model can not only represent the attenuation and constant stage of feature parameters but also reflect the nonlinear increase stage of feature parameters
2. The change curve of input image size *W* has obvious fluctuation characteristic, while the curve corresponding to convolution size *F*, image filling edge *P*, and step size *S* is basically the same. It shows that these three parameters have basically the same influence on the graph output, and the graph size *W* has the largest influence. Therefore, we need to consider the influence of various factors comprehensively when selecting different parameters
3. The output image size after pooling can be divided into two different change stages according to different influencing factors. Relevant studies show that parameter *I* has a positive influence on the output size, while parameter *P*_*s*_ has a negative influence on the output value *O*

## Figures and Tables

**Figure 1:** Performance comparison diagram of two models.

**Figure 2:** MP model.

**Figure 3:** Contour variation diagram of offset term.

**Figure 4:** Gradient diagram of different functions.

**Figure 5:** Development history of convolutional neural network.

**Figure 6:** Influence curve of different coefficients on convolution layer.

**Figure 7:** Influence of size and channel on the number of parameters.

**Figure 8:** Image size output value after pooling.

**Figure 9:** Proportion of predicted value of parameter *i* to different samples.

**Figure 10:** Distribution diagram of different characteristic indexes.

**Figure 11:** Cardio-cerebrovascular metabolic flow chart based on convolutional neural network.

**Figure 12:** Summary diagram of metabolic characteristics of cardiovascular and cerebrovascular diseases based on convolutional neural network.

**Figure 13:** Model prediction diagram.

## Data Availability

The experimental data used to support the findings of this study are available from the corresponding author upon request.
